# Silencing *MYOT* Expression May Inhibit Autophagy in Human Skeletal Muscle Cells

**DOI:** 10.1155/2023/3350685

**Published:** 2023-02-02

**Authors:** Zhao-Jing Lin, Jun-Mei Xu, He-Yu Ji, Ya-Qing Jiang, Jun Su, Liang-Liang Fan, Rong Yu

**Affiliations:** ^1^Department of Anesthesiology, The Second Xiangya Hospital of Central South University, Changsha, 410011 Hunan Province, China; ^2^Department of Cell Biology, School of Life Sciences, Central South University, Changsha 410013, China

## Abstract

Muscle diseases are closely related to autophagy disorders. Studies of autophagy inhibition indicated the importance of autophagy in muscle regeneration, while activation of autophagy can restore muscle function in some myopathies. Previous studies have revealed that mutations in the *MYOT* gene may lead to several kinds of hereditary myopathies. However, whether the autophagy played a crucial role in hereditary myopathy caused by *MYOT* mutations was still not clear. In this study, we established the *MYOT* knockdown human skeletal muscle cell models (HSkMCs) by small interfering RNA. Real-time PCR and Western blot studies found that the expression of *p62* and *LC3B-II* was decreased dramatically, which suggested that silencing *MYOT* expression may regulate the autophagy in HSkMCs. Further immunofluorescence study on Ad-mCherry-GFP-LC3B adenovirus transfection and monodansylcadaverine (MDC) staining revealed that knocking down the expression of *MYOT* may inhibit the autophagy. Next, we used the autophagy inducer Earle's balanced salt solution (EBSS) and late-autophagy inhibitor bafilomycin A1 (BAF A1) to treat the HSkMCs, respectively, and found that silencing *MYOT* expression can inhibit the activation of autophagy by EBSS and aggravate the inhibition of autophagy by BAF A1. Finally, we also found that silencing *MYOT* expression can downregulate the expression of ATG7 and ATG5, two important autophagy regulatory molecules. Hence, our study may first reveal that knocking down the expression of *MYOT* may inhibit the autophagy. Hereditary myopathies caused by *MYOT* mutations may partly result from the inhibition of autophagy in HSkMCs.

## 1. Introduction

Skeletal muscle cells are composed of hundreds of myofibrils. A section of myofibrils between two adjacent Z-discs is called a sarcomere. A sarcomere is a basic unit of not only skeletal muscle fiber structure but also muscle cell contraction and relaxation. For decades, Z-discs were thought to play a single and specific role: maintain myofibril architecture. This view has changed dramatically in the past decade, and now, Z-discs are recognized as important hubs of signaling, mechanosensing, and mechanotransduction, playing novel roles in protein turnover and autophagy [1, 2].

Myotilin is a component of Z-disc proteins with a molecular weight of 57 kDa and is encoded by the *MYOT* gene on chromosome 5q31.2. The *MYOT* gene contains 10 exons, encodes 498 amino acids, and is highly expressed in skeletal muscle and moderately expressed in the heart. Myotilin crosslinks actin filaments [3] by binding to *α*-actinin [3, 4] and filamin C [5, 6]. Myotilin stabilizes and anchors thin filaments to Z-discs during myofibril formation and plays an important role in sarcomere assembly [3, 4, 7]. The resulting structure maintains the integrity of skeletal muscle cells and their contractile function [5]. *MYOT* gene mutations can cause slowly progressive and late-onset myofibrillar myopathies, limb-girdle muscular dystrophy type 1A (LGMD 1A), myofibrillar myopathy (MFM), or spheroid body myopathy [8–10].

Skeletal muscle tissue plays a significant role in the normal life activities of human body, and the stability of the skeletal muscle autophagy level is crucial for the maintenance of skeletal muscle mass. Skeletal muscle autophagy level changes due to various reasons; it may lead to muscle tissue diseases. As part of the Z-disc protein, MYOT (myotilin) could participate in autophagy maintenance in the skeletal muscle. Although myotilin plays important roles in a skeletal muscle structure and function, few studies have focused on the mechanism of myotilin deficiency. In this study, we aim to explore the role of *MYOT* in autophagy in human skeletal muscle cells (HSkMCs).

## 2. Materials and Methods

### 2.1. Cell Culture

The HSkMC line (cat#: BFN60804003, BFB Life Sciences, China) was cultured in DMEM (cat#: C11995500BT, Gibco, USA) with 10% fetal bovine serum (cat#: SFBS, BOVOGEN, Australia) and 50 units/ml penicillin with 50 *μ*g/ml streptomycin (cat#: SV30010, HyClone, USA). The medium was changed, or the cells were passaged every 2-3 days. The cells were maintained in a cell incubator (Thermo Fisher, USA) under humidified conditions with 5% CO_2_ at 37°C.

Earle's balanced salt solution (EBSS, cat#: C0213, Beyotime Biotechnology, China) and 100 nM bafilomycin A1 (BAF A1, cat#: 54645S, CST, USA) were served as the autophagy inducer and autophagy inhibitor in this study.

### 2.2. Construction of Small Interfering RNAs (siRNAs) to Specifically Silence the MYOT Gene

*MYOT* siRNAs were designed according to the mRNA sequence of the human *MYOT* gene (NM_001135940.2.) as documented in the Human GenBank database. The three siRNA sequences were si-*MYOT*(1) (5′-GCACCAATGTTTATCTACAdTdT-3′, 5′-TGTAGATAAACATTGGTGCdTdT-3′, cat#: stB0009006A-1-5, RiboBio, China), si-*MYOT*(2) (5′-GCAAGTTCCTACATCACAAdTdT-3′, 5′-TTGTGATGTAGGAACTTGCdTdT-3′, cat#: stB0009006B-1-5, RiboBio, China), and si-*MYOT*(3) (5′-CAGAGAACATGTCGATTGAdTdT-3′, 5′-TCAATCGACATGTTCTCTGdTdT-3′, cat#: stB0009006C-1-5, RiboBio, China). In addition, a scrambled siRNA was used as the negative control (si-control) (cat#: siN0000001-1-5, RiboBio, China). All the siRNA sequences were purchased from Guangzhou RiboBio Co., Ltd.

### 2.3. Establishment of the MYOT-Knockdown Cell Model

Cells were seeded in 6- or 24-well plates at a density of 1.5 × 10^5^ cells/ml in a complete medium without penicillin–streptomycin. The next day, when the cells reached 80% confluence, siRNAs were transfected with riboFECT CP Transfection Kit (166T) (cat#: C10511-05, RiboBio, China) at a concentration of 30 nM siRNA following the manufacturer's directions. Cell samples were harvested 48 hours after transfection. Cells transfected with si-control were the negative controls.

### 2.4. Cell Viability Detection

The Cell Counting Kit-8 (CCK8, CA1210, Solarbio, China) was used to detect the cell viability. Cells were seeded in 96-well plates at a density of 1.5 × 10^5^ cells/ml. When the cells reached 80% confluence, we then treated the cells with 30 nM siRNA. 48 hours later, 10 *μ*l CCK8 solution was added into the well and incubated in 37°C incubator for 4 hours. Finally, the absorbance was detected at 450 nm in a microplate reader (Thermo Scientific).

### 2.5. Real-Time PCR

Total RNA was extracted by TRIzol reagent (cat#: 15596-026, Invitrogen, USA) and reverse transcribed with a cDNA synthesis kit (cat#: QP056, GeneCopoeia, China) to obtain cDNA. Real-time qPCRs were carried out in Fast 7500 Real-Time PCR Systems (Applied Biosystems) using Maxima SYBR Green/ROX qPCR Master Mix (2×) (Thermo Fisher Scientific, #K0221). The reaction conditions were as follows: predenaturation at 95°C for 30 s, denaturation at 95°C for 10 s, and annealing and extension at 60°C for 30 s in a total of 40 cycles.

*GAPDH* was selected as the endogenous control gene. Human *MYOT* primers (forward, 5′-GGGTCTTCATTCACTCATCTTTGA-3′, and reverse, 5′-GGTGGCTTCTCCTGCTCTAT-3′), human *GAPDH* primers (forward, 5′-CCCTTCATTGACCTCAACTACA-3′, and reverse, 5′-ATGACAAGCTTCCCGTTCTC-3′), and human *SQSTM1/P62* primers (forward, 5′-TGATTGAGTCCCTCTCCCAGATGC-3′, and reverse, 5′-CCGCTCCGATGTCATAGTTCTTGG-3′) were used. The primers were synthesized by Sangon Biotech Co. Ltd. (Shanghai, China). The 2^-△△Ct^ method was used to calculate the relative expression levels of genes and report these levels as fold changes.

### 2.6. Western Blotting

The cells were harvested, and the total protein was extracted on ice with M-PER Mammalian Protein Extraction Reagent (cat#:78505, Thermo, USA). Fifteen micrograms of protein was separated by SDS–PAGE and transferred to PVDF membranes (cat#: ISEQ00010, Millipore, USA). After blocking in 5% fat-free milk in a TBST solution, the membranes were incubated overnight at 4°C with the following primary antibodies: anti-MYOT (1 : 500, cat#: a6439, ABclonal, Wuhan, China), anti-GAPDH (1 : 5000, cat#: 60004-1-Ig Proteintech, USA), anti-LC3B (1 : 1000, cat#: ab192890, Abcam, USA), anti-SQSTM1/p62 (1 : 1000, cat#: sc-28359, Santa Cruz Biotechnology, USA), anti-ATG5 (1 : 1000, cat#: 12994, CST, USA), anti-ATG7 (1 : 1000, cat#: 8558, CST, USA), and anti-ATG12 (1 : 1000, cat#: 4180, CST, USA). The next day, the membranes were incubated for 1 hour at room temperature with the corresponding secondary antibodies. The protein bands were visualized with Western Bright enhanced chemiluminescence horseradish peroxidase (ECL HRP) substrate (cat#: K-12045-D50, Advansta, USA). The protein bands were photographed with a Clinx Science Instrument, and the data were analyzed with ImageJ software.

### 2.7. Immunofluorescence

HSkMCs were seeded at a density of 1.5 × 10^5^ cells/ml on a cover glass (cat#: 801010, NEST, China) in 24-well plates, and 24 hours later, siRNAs were transfected into these cells. The cells were harvested 48 hours after siRNA transfection. They were washed in PBS three times, fixed in 4% paraformaldehyde for 15 minutes, permeabilized with 0.3% Triton X-100 for 3 minutes, and blocked with 1% bovine serum albumin (BSA) in PBS for 40 minutes at room temperature. Then, the primary antibody was added and incubated with the cells for 1 hour at room temperature. After washing with PBS, the cells were sequentially incubated with the corresponding secondary antibody for 1 hour. Phalloidin was used for cytoskeleton staining, and DAPI was used for nuclear staining. The pictures were captured under a fluorescence microscope (OLYMPUS).

### 2.8. Ad-mCherry-GFP-LC3B Adenovirus Transfection

The Ad-mCherry-GFP-LC3B adenovirus was purchase from Beyotime (C3011, Beyotime Biotechnology, China). HSkMCs were seeded into 12-well plates. When the cells reached 80% confluence, adenovirus Ad-mCherry-GFP-LC3B was added to the cells for 24 h. Then, culture medium containing the virus was removed and replaced with normal medium for 24 h. The immunofluorescence study refers to abovementioned methods.

### 2.9. Monodansylcadaverine (MDC) Staining

A proper amount of MDC (1000x) was diluted to MDC (1X) by assay buffer at a ratio of 1 : 1000 using Autophagy Staining Assay Kit with MDC (cat#: C3019S, Beyotime Biotechnology, China). The medium in the 24-well plates was replaced with MDC (1x), and the cells were incubated in a cell incubator for 30 minutes away from the light. Then, the cells were washed three times with assay buffer (1×). 250 *μ*l of assay buffer (1×) was added and placed the samples under a fluorescence microscope. The green fluorescence distribution was observed and recorded under a fluorescence microscope (OLYMPUS).

### 2.10. Statistical Analysis

Statistical analysis was performed with GraphPad Prism v6.0 software (GraphPad Software, Inc., La Jolla, CA, USA). The results represent the mean ± SD from at least three independent experiments. Two-tailed Student's *t*-tests based on ANOVA were used for 2-group comparisons. ^∗^ means *P* < 0.05, ^∗∗^ means *P* < 0.01, ^∗∗∗^ means *P* < 0.001, and ns means no significance.

## 3. Results

### 3.1. Silencing MYOT Expression Reduce the Expression of P62 and LC3B-II

Three siRNA sequences which may silence the expression of *MYOT* were prepared in this study. We then applied the real-time PCR to screen the most effective one and found that the third siRNA which is named si-*MYOT*(3) showed the best silence ability (Figure 1(a)). Next, we also screened the effective concentration of the third siRNA and found that 30 nM may be an appropriate concentration for si-*MYOT*(3) (Figure 1(b)). The Western blot further validated the reduction of MYOT in HSkMCs treated with 30 nm si-*MYOT*(3) (Figures 1(c) and 1(d)). The CCK8 study revealed that the silencing *MYOT* expression did not affect the cell viability (Figure 1(e)). Hence, we established an effective HSkMC model with silencing *MYOT* expression. The 30 nM si-*MYOT*(3) was applied in the following studies.

Next, we detected the expression of p62 by real-time PCR and found that the mRNA levels were decreased in HSkMCs transfected with si-*MYOT* (Figure 2(a)). Further Western blot validated that the expression of p62 in the si-*MYOT* group was obviously lower than that in the si-control group (Figures 2(b) and 2(c)). Then, we detected the LC3B-II levels and found that the expression of LC3B-II in the si-*MYOT* group was also reduced dramatically compared to the si-control group (Figures 2(d) and 2(e)). Previous studies have demonstrated that the tendency of p62 and LC3B-II should be opposite during autophagy [11]. Here, in our study, both p62 and LC3B-II were decreased when silencing the *MYOT* expression. Our study indicated a strong correlation between decreased MYOT levels and autophagy.

### 3.2. Silencing MYOT Expression Can Inhibit Autophagy

In order to confirm silencing *MYOT* expression can inhibit autophagy or activate autophagy, we then perform the immunofluorescence study and found that the expression of LC3B was obviously decreased in the si-*MYOT* group (Figure 3(a)). The Ad-mCherry-GFP-LC3B adenovirus transfection study further confirmed that in the si-*MYOT* group, the HSkMCs showed the diffuse yellow distribution, which indicated that the autophagy was inhibited (Figure 3(b)). Simultaneously, MDC staining also revealed that the green fluorescence levels were decreased in the si-*MYOT* group, which indicated that the number of autophagosome in the si-*MYOT* group was less than the si-control group (Figure 3(c)). All these immunofluorescence studies suggested that silencing *MYOT* expression may inhibit autophagy.

### 3.3. Silencing MYOT Expression Can Inhibit the Activation of Autophagy by EBSS

Next, the HSkMCs were treated with EBSS to activate the autophagy, and the Ad-mCherry-GFP-LC3B adenovirus transfection study showed that the diffuse yellow distribution was presented in the si-*MYOT* group after EBSS treatment, which indicated that silencing *MYOT* expression can inhibit the EBSS-induced autophagy (Figure 4(a)). Meanwhile, the MDC staining revealed that the green fluorescence levels in the si-control group were much higher than those in the si-*MYOT* group after EBSS treatment, which suggested that silencing *MYOT* expression can reduce the number of autophagosome induced by EBSS (Figure 4(b)). Both studies proved that silencing *MYOT* expression can inhibit the activating of autophagy by EBSS.

### 3.4. Silencing MYOT Expression Can Aggravate the Inhibition of Autophagy by BAF A1

We then applied BAF A1 to treat the HSkMCs to inhibit autophagy. An immunofluorescence study showed that the expression of LC3B in the si-*MYOT* group was lower than that in the si-control group after BAF A1 treatment, which indicated that the number of autophagosome was decreased when silencing *MYOT* expression (Figure 5(a)). The Ad-mCherry-GFP-LC3B adenovirus transfection study showed that both the si-control group and the si-*MYOT* group showed the diffuse yellow distribution after BAF A1 treatment (Figure 5(b)). However, the MDC staining presented that the green fluorescence levels in the si-control group were higher than those in the si-*MYOT* group after BAF A1 treatment, which suggested that silencing *MYOT* expression can further reduce the number of autophagosome (Figure 5(c)). These observations suggested that silencing *MYOT* expression can aggravate the inhibition of autophagy by BAF A1.

### 3.5. Silencing MYOT Expression May Reduce the Expression of ATG7 and ATG5

Finally, we employed Western blot to detect the expression of LC3B-II, ATG5, ATG7, and ATG 12 in HSkMCs treated with BAF A1 and/or transfected with si-*MYOT*. The results showed that compared to that in the si-control group, the protein expression level of LC3B-II in the si-*MYOT* group was decreased (Figures 6(a) and 6(b)). Compared to that in the si-control+BAF A1 group, the expression level of LC3B-II protein in the si-*MYOT*+BAF A1 group was decreased (Figures 6(a) and 6(b)). Compared to that in the si-control group, the ATG7 protein expression level in the si-*MYOT* group was significantly decreased (Figures 6(a) and 6(b)). Moreover, the ATG5 and ATG12 protein levels were also analyzed, and the expression of the ATG5 protein in the si-*MYOT*+BAF A1 group was decreased compared to that in the si-control+BAF A1 group (Figures 6(a) and 6(b)). These studies further confirmed that silencing the *MYOT* expression can inhibit autophagy.

## 4. Discussion

*MYOT* mutations mainly manifest in myopathies, which are referred to as “myotilinopathies” [12]. Myotilinopathy variants often lead to structural changes in Z-discs and the formation of polymorphic aggregates [10, 13]. Myotilinopathy is often negatively affected by delayed diagnosis, misdiagnosis, and lack of effective treatment [14]. Searching for new targets closely related to the occurrence and development of a myotilinopathy and studying the molecular mechanism of target biological functions in skeletal muscle cells may lead to possible ideas and a theoretical basis for the early myotilinopathy diagnosis and clinical treatment.

Autophagy is a dynamic process that requires the formation of phagocytic vesicles, followed by the formation of autophagosomes, which fuse with lysosomes to become autophagolysosomes and, ultimately, autophagolysosome degradation [15]. To date, three major forms of autophagy have been described: macroautophagy, chaperone-mediated autophagy, and microautophagy [16–18]. Macroautophagy is typically called autophagy, which is closely related to myopathy. During macroautophagy (hereafter, autophagy), cytosolic components are surrounded by double-membrane structures that form the autophagosome, which then fuse with lysosomes, which degrade the autophagosome-sequestered contents [19].

Our study explored that knocking down the expression of MYOT in HSkMCs may change the autophagic flux. After specifically knocking down the expression of *MYOT*, we found that the p62 levels were decreased, and the LC3B-II levels were also reduced, which was not consistent with previous studies in autophagy that indicated that the tendency of p62 and LC3B-II should be opposite during autophagy [11]. Generally, the increasing of LC3B-II or the conversion of LC3B-I to LC3B-II were represented to the initiation of autophagy [20]. The reduction of LC3B-II has been proved to be the inhibition of autophagy [21]. In this study, we detected the reduction of LC3B-II and also applied the immunofluorescence study, the Ad-mCherry-GFP-LC3B adenovirus transfection study, and MDC staining to further confirm that silencing the expression of MYOT may inhibit the autophagy. Simultaneously, previous studies have revealed that the expression of ATG7, ATG5, and ATG12 was also related to autophagy [22]. Hence, we also detected the expression of these three proteins and found that the expression of ATG7 and ATG5 was decreased in the si-MYOT group or si-MYOT+BAF A1 group, which further confirmed that the autophagy was inhibited in the si-MYOT group. We may first establish the relationship between MYOT and autophagy, which may provide news perspectives between MYOT and myofibrillar myopathies.

In several muscle diseases, alterations to autophagic flux have been reported to contribute to pathological mechanisms of action [23]. Autophagy inhibition was first demonstrated with collagen VI-knockout mice that had been used to establish a congenital muscular dystrophy model [24]. The study of autophagic flux in the collagen VI-knockout mice was made easier by the many similarities in the muscle phenotype of ATG7-knockout mice and collagen VI-knockout mice; the results showed an autophagy induction defect that ultimately led to abnormal clearance of damaged organelles, which was accompanied by oxidative stress, fiber atrophy, fiber cell apoptosis, and muscle degeneration [24]. Subsequently, a partial failure of autophagy induction has been found in *MDX*-mutant mice, models of Duchenne muscular dystrophy [25], confirming the role played by autophagy-induced defects in the pathogenesis of multiple muscular dystrophies. More importantly, researchers have found that autophagy induction by starvation or a low-protein diet resulted in anatomical and functional enhancements in two models of dystrophy [24, 25], suggesting that autophagy-induced defects in muscular dystrophy are biologically significant.

## 5. Conclusions

In conclusion, our study may first reveal that knocking down the expression of *MYOT* may inhibit the autophagy. Hereditary myopathies caused by *MYOT* mutations may partly result from the inhibition of autophagy in HSkMCs.

## Figures and Tables

**Figure 1:** The *MYOT* was knocked down effectively by siRNA in HSkMCs. (a) Real-time PCR detected the mRNA levels of the *MYOT* in HSkMCs transfected with three siRNAs, respectively. (b) Real-time PCR detected the mRNA levels of the *MYOT* in HSkMCs transfected with different concentrations of si-*MYOT*(3). (c) Western blot detected the protein levels of *MYOT* in HSkMCs transfected with 30 nm si-*MYOT*(3). (d) The statistical results of *MYOT*. (e) CCK8 detected the cell viability in the WT, si-control, and si-*MYOT* groups.

**Figure 2:** Silencing *MYOT* expression reduces the expression of P62 and LC3B-II. (a) Real-time PCR detected the mRNA levels of p62 in HSkMCs transfected with si-*MYOT*. (b) Western blot detected the protein levels of p62 in HSkMCs with *MYOT* knocking down. (c) The statistical results of p62. (d) Western blot detected the protein levels of LC3B-II in HSkMCs transfected with si-*MYOT*. (e) The statistical results of LC3B-II.

**Figure 3:** Silencing *MYOT* expression can inhibit autophagy. (a) Immunofluorescence detected the expression of LC3B and Phalloidin in HSkMCs transfected with si-*MYOT*. (b) The Ad-mCherry-GFP-LC3B adenovirus transfection study showed the autophagy levels of HSkMCs transfected with si-*MYOT*. (c) MDC staining showed the autophagy levels of HSkMCs transfected with si-*MYOT*.

**Figure 4:** Silencing *MYOT* expression can inhibit the activation of autophagy by EBSS. (a) The Ad-mCherry-GFP-LC3B adenovirus transfection study showed the autophagy levels activated by EBSS in HSkMCs transfected with si-*MYOT*. (b) MDC staining showed the autophagy levels activated by EBSS in HSkMCs transfected with si-*MYOT*.

**Figure 5:** Silencing *MYOT* expression can aggravate the inhibition of autophagy by BAF A1. (a) Immunofluorescence detected the expression of LC3B and Phalloidin in HSkMCs treated with BAF A1 and transfected with si-*MYOT*. (b) The Ad-mCherry-GFP-LC3B adenovirus transfection study showed the autophagy levels inhibited by BAF A1 in HSkMCs transfected with si-*MYOT*. (c) MDC staining showed the autophagy levels inhibited by BAF A1 in HSkMCs transfected with si-*MYOT*.

**Figure 6:** Silencing *MYOT* expression may reduce the expression of ATG7 and ATG5. (a) Western blot analyzed the expression of LC3B-II, ATG7, ATG5, and ATG 12 in HSkMCs treated with BAF A1 or transfected with si-*MYOT*. (b) The statistical results of LC3B-II, ATG7, ATG5, and ATG12.

## Data Availability

The datasets used and/or analyzed during the current study are available from the corresponding author upon reasonable request.
